The article "Application Effect of Somatostatin Combined with Transnasal Ileus Catheterization in Patients with Acute Intestinal Obstruction and Advanced Gastric Cancer" was retracted in 2023. Reasons: signs of a paper mill; compromised peer review; unreliable results or conclusions.

# Application Effect of Somatostatin Combined with Transnasal Ileus Catheterization in Patients with Acute Intestinal Obstruction and Advanced Gastric Cancer

**DOI:** 10.1155/2022/9747880

**Published:** 2022-06-11

**Authors:** Zhenlu Li, Zhen Liu, Zongping Yu

**Affiliations:** Department of Emergency Surgery, The Affiliated Hospital of Qingdao University, Qingdao 266003, China

## Abstract

*Objective*: To explore the application of somatostatin combined with nasal plug catheterization in patients with advanced gastric cancer and acute intestinal obstruction. *Methods*. This study included 94 cases of patients with acute intestinal obstruction and advanced gastric cancer, and according to the length of hospital stay, the patients were randomly divided into two groups: the control group and the study group, with 47 cases in each group. Based on the observations made by the team in the control group given somatostatin combined treatment, we observed two groups of patients with gastrointestinal function, serum index, quality of life, therapeutic effect, and adverse reactions. *Results*. Abdominal distention, abdominal pain duration, and normal exhaust time were significantly shorter in the study group than in the control group. The study group was higher than the control group in terms of gastrointestinal decompression volume, drainage volume, and abdominal circumference reduction within 24 hours (*P* < 0.05). After treatment, the levels of CRP, IgA, LPS, and FABP were lower than before, and the levels of CRP, IgA, LPS, and FABP in the former group were much lower than those in the latter group (*P* < 0.05). Compared with before treatment, the former GIQLI scale score was significantly higher than the latter (*P* < 0.05). After treatment, the efficiency is much higher than the latter (*P* < 0.05). After treatment, the former significantly lowers the incidence of postoperative complications of the latter (*P* < 0.05). *Conclusion*. For patients with advanced gastric cancer and acute intestinal obstruction, it is safe and feasible to use somatostatin combined with transnasal intestinal obstruction catheterization to restore gastrointestinal function, improve inflammatory response, and promote the improvement of quality of life with high safety and feasibility.

## 1. Introduction

Gastric cancer refers to malignant tumors of gastric mucosal epithelial tissue [1]. It is one of the cancers with the highest incidence in all mankind. The incidence of cancer increases with age, mainly in middle-aged and elderly men, and the mortality rate accounts for about 25% of cancer deaths, posing a serious threat to human life and health. The incidence of gastric cancer is affected by factors such as bad diet and living environment, heredity, and pathogenic bacterial infection. Most of them are in the middle and late stages of endoscopic examination, which are manifested as upper abdominal tenderness, digestive system disorders, and hematemesis [2, 3]. Clinical treatment for advanced gastric cancer patients to take surgical treatment, the treatment effect is remarkable. However, the distant metastasis of cancer cells and gastrointestinal injury are prone to causing acute intestinal obstruction, which affects treatment and prognosis [4]. Acute ileus is a mechanical blockage of intestinal contents, resulting in abdominal distention, acid-base electrolyte balance, and vomiting. If active and effective treatment is not adopted, life safety is often critical [5,6].

Clinically, individualized treatment schemes are often adopted according to the cause, location, degree, and systemic physiological disorder of intestinal obstruction, such as regulating water, electrolyte, acid-base balance, and gastrointestinal decompression. Treatment that ameliorates physiological disorders is difficult to cure completely. Gastrointestinal decompression is usually accomplished through catheter placement, which can effectively discharge the gas and liquid in the digestive system. It reduces and twists intestinal loops, and relieves blood circulation and edema in the intestinal wall. However, it can cause respiratory circulation blockage, resulting in lung infection and so on. In addition, traditional implantation has limited decompression sites, limited effect on reducing intraabdominal pressure, and unsatisfactory therapeutic effect [7–9]. In recent years, transnasal intestinal obstruction catheterization has been widely used in clinical practice, which can ensure the total decompression of the small intestine and effectively relieve clinical symptoms. Patients with acute intestinal obstruction and advanced gastric cancer who were hospitalized between May 2020 and May 2021 were enrolled in the study. The effects of single intervention and combined intervention of somatostatin on gastrointestinal function, serum indexes, quality of life, efficacy, and adverse reactions of patients with nasal obstruction catheterization were investigated. The report follows.

## 2. Data and Methods

### 2.1. General Information

The study included 94 patients with acute ileus and advanced gastric cancer hospitalized between May 2020 and May 2021. We randomly divided 47 patients into control group and study group according to the length of hospital stay. Control group comprised 28 cases (male) and 19 cases (female). The mean duration of gastric cancer was 5.29 ± 1.37 months, and the mean duration of ileus was 2.67 ± 0.72 days. There were 27 males and 20 females in the observation group. The average age was 50.03 ± 5.35 from 39 to 72 years old. The mean course of gastric cancer was 5.30 ± 1.36 months, and the mean course of ileus was 2.69 ± 0.70 days. The basic data were similar between the two groups and had no statistical significance (*P* > 0.05), indicating comparability. The control group adopted the treatment of nasal obstruction, while the study group was treated by somatostatin combined. This study was approved by our hospital medical ethics committee.

### 2.2. Inclusion and Exclusion Criteria

  Inclusion criteria [10]: ① in line with the diagnostic criteria of acute intestinal obstruction with advanced gastric cancer in the emergency, differential diagnosis and treatment guidelines for acute intestinal obstruction and the 2018 edition of Gastric Cancer Diagnosis and Treatment Guidelines; ② acute intestinal obstruction with advanced gastric cancer were diagnosed by fibercolonoscopy, gastroscopy, and pathological biopsy; (3) clinical manifestations of postoperative abdominal pain, vomiting, abnormal defecation and exhaust, gastrointestinal tenderness and voiced sound; (4) recent history of abdominal surgery; ⑤ no cognitive and mental disorders, with normal communication skills; and ⑥ the subjects knew the content of the study and signed informed consent according to their wishes.
  Exclusion criteria [11]: ① patients with severe organ function or other malignant tumors; ② estimated survival time ≤1 month; ③ with other abdominal and digestive system inflammation or serious diseases; ④ with abnormal immune system and coagulation function; ⑤ incomplete clinical data; and ⑥ poor compliance.

### 2.3. Research Methods

After admission, all patients filled in their basic personal information, underwent abdominal CT, endoscopy, and other imaging examinations, and evaluated the corresponding scales and indicators. After cancer treatment, basic intervention was given, including gastrointestinal decompression, nutritional support, maintenance of water, electrolyte and acid-base balance, health education, acid inhibition, antiinfection, and precautions. Patients' vital signs and electrocardiogram, attention, and prevention of adverse events or complications were closely monitored. Patients were informed about fasting before surgery to improve the pressure in the intestinal cavity. The control group was given the treatment of nasal intestinal obstruction catheter implantation: a transnasal intestinal obstruction catheter 300 cm long and a guidewire 350 cm long containing two sacs and three chambers. The patient was instructed to take the semidecubitus position, the anterior capsule of the catheter was filled with distilled water and coated with lubricant, and the guidewire was reserved in the catheter. Note that the guidewire is inside the catheter. With the assistance of gastroscopy, the catheter is placed into the upper jejunum through the greater curvature of the stomach, during which residual fluid of the upper digestive tract is absorbed. Exit the gastroscope and extract the guidewire. The depth of the catheter is about 50∼60 cm. Ensure that the catheter is kept at a certain distance from the obstruction position, the outer segment of the catheter is connected to the negative pressure suction device, the inner tube is responsible for adding water to decompress, and the outer tube is responsible for sucking gastrointestinal contents. Instruct the patient to take the catheter position, pay attention to cleaning the catheter every day, and maintain the drainage tube smooth. When normal exhaust, eating and symptoms improve, the catheter can be removed. If the situation is not improved or repeated, a contrast agent can be injected to observe intestinal obstruction. The study group was given somatostatin combination therapy based on the control group: intravenous somatostatin (Beijing SL Pharmaceutical Co., Ltd., National Drug Approval H20054016, specification: 3 mg*∗*5 tablets/box) and 0.6 mg somatostatin +0.9% normal saline 100 mL before use. The flow rate was controlled at 0.25 mg/h, and the infusion was continued for 24–48 h. When the interval between two transfusions is 3 to 5 minutes, 0.25 mg should be intravenously injected. In the process of treatment, the dosage may be adjusted according to the patients' symptoms and exhaust conditions. The normal treatment time is 5 days. Try not to exceed 2 weeks.

### 2.4. Observation Indicators

① Degree of gastrointestinal function improvement: duration of abdominal distention and pain, normal exhaust time, gastrointestinal decompression volume, drainage volume, and abdominal circumference reduction within 24 hours were recorded in two groups. ② Serum-related index determination: 3 ml of fasting venous blood was drawn from patients before and after treatment. After centrifugation and standing treatment, the supernatant was taken and stored at −80°C for further examination. C-reactive protein (CRP) was detected by a reaction analyzer (Beckman Coulter Trading Co., LTD. DxH 600). The levels of immunoglobulin A (IgA), lipase (LPS), and fatty acid-binding protein (FABP) were detected by flow cytometry and enzyme-linked immunoassay. The kit is provided by Shanghai Enzyme Linked Biotechnology Co., LTD., and is operated in strict accordance with the kit testing standards. ③ Comparison of quality of Life: Gastrointestinal Quality of Life Index [12] (GIQLI) was used to measure the quality of life of patients before and after treatment. There are 36 items on the scale, and the scoring method is 0 to 5, ranging from “all the time” to “never,” including five dimensions of conscious behavior, physiological state, psychological emotion, social role, and special situation. The score indicates a good quality of life. (4) Clinical treatment effect: according to the clinical symptoms and vital signs of patients in each group, the treatment effect of patients in the two groups was evaluated, and recovered: abdominal distention, abdominal pain and other symptoms disappeared, exhaust and defecation, serum indicators and other normal, daily life and work had no impact; effective: abdominal distention, abdominal pain, and other symptoms have been alleviated, exhaust defecation, serum indicators have been improved; invalid: no change or aggravation of clinical symptoms and vital signs. Clinical effectiveness = (cure + effective) cases/total number of cases by 100%. ⑤ The adverse reactions, including infection, allergic reaction, nausea and vomiting, dizziness, and effusion, were observed and recorded during the 1 month follow-up.

### 2.5. Statistical Treatment

Using the SPSS 24.0 statistical software. To conform to the normal distribution of measurement data with $\bar{x}$ ± *S*, comparison between groups by *t*-test. Statistics of the number of cases (*n*) and the percentage (%), the comparison between groups by chi-square test to *P* < 0.05 for the difference was statistically significant.

## 3. Results

### 3.1. Comparison of Improvement Degree of Gastrointestinal Function

Results show that the duration of the abdominal distension and abdominal pain in the team is shorter than that in the control group, and gastrointestinal decompression and drainage flow and reduce abdominal circumference team within 24 hours is higher than that in the control group, see Table 1.

### 3.2. Comparison of Serum-Related Indicators

Results show that the regarding energy metabolism index in both groups before treatment, there was no statistically significant difference (*P* < 0.05). After treatment, the levels of two groups of patients with CRP, IgA, LPS, and FABP were lower than those before treatment, and the differences were statistically significant (*P* < 0.05). The CRP, IgA, LPS, and FABP levels of the former were much lower than those of the latter; see Table 2 and Figure 1.

### 3.3. Comparison of Quality of Life

The results show that between the two groups of patients before treatment GIQLI score comparison, there was no statistically significant difference (*P* > 0.05); after treatment, the scores of consciousness, behavior, physiological state, psychological emotion, social role, Figure 2special situation and other aspects of patients in each group were changed, and the differences were statistically significant (*P* < 0.05). GIQLI: the former scale score was much higher than that of the latter, as shown in Table 3 and.

### 3.4. Treatment Effect Comparison

Results show that the effective rate of 95.74% was higher than 87.23% of the control group, as shown in Table 4.

### 3.5. Comparison of Incidence of Adverse Reactions

According to the results, the team incidence of postoperative complications (8.51%) was much lower than the control group (14.89%), as shown in Table 5.

## 4. Discussion

With the change in dietary habits and environments, the incidence and mortality of gastric cancer have increased every year. Among these, acute intestinal obstruction, as one of the serious complications after gastric cancer surgery, has adverse effects on the treatment and prognosis. For patients with advanced gastric cancer, distant metastasis of cancer tissues and cells is easy to occur, resulting in a large range of lymph node dissection and large gastrointestinal stimulation during gastric cancer surgery. After surgery, due to the decrease of gastrointestinal motion amplitude and degree, an internal hernia or intestinal loop is generated between the intestines, which eventually leads to acute intestinal obstruction [13]. Clinical treatment of intestinal obstruction is mostly symptomatic treatment and surgical treatment, among which surgical treatment is more stimulating and damaging to the body and prone to postoperative adverse events [14]. Therefore, the selection of safe and effective treatment means is the focus of the gastroenterology department. Transnasal intestinal obstruction catheterization can effectively control intestinal spasm and intraabdominal pressure, improve intestinal circulation and water and electrolyte balance, and relieve clinical symptoms. Somatostatin, as an important inhibiting hormone in the gastrointestinal tract, can effectively inhibit the secretion of gastric and digestive juices. At the same time, it can also improve gastrointestinal bleeding and edema symptoms, affect digestive system movement, blood flow, etc., with significant effects [15,16]. At home and abroad, the pathogenesis and surgical treatment of acute intestinal obstruction are often concerned, while less attention is paid to the influence of somatostatin combined with transnasal intestinal obstruction catheter insertion [17,18]. In this study, somatostatin combined with transnasal intestinal obstruction catheterization was used to treat acute intestinal obstruction with advanced gastric cancer, which can effectively relieve symptoms such as abdominal distention and abdominal pain, improve gastrointestinal internal environment and quality of life, and improve the therapeutic effect.

Extrusion of abdominal contents and prolonged exposure during surgery will cause local stress response, which will lead to abnormal expression of inflammatory factors and increase the difficulty of treatment. CRP, as an acute reactive factor, can sensitively reflect the degree of infection and treatment effect. As an immune effector with antibody activity in the body, IgA can participate in and regulate the humoral immune system. LPS can promote the synthesis and secretion of inflammatory factors and then induce systemic inflammation. As a specific and sensitive indicator of gastric mucosal ischemia, FABP can reflect the condition of gastric mucosal ischemia and damage [19,20]. Lin et al. [21] used transnasal intestinal obstruction catheterization to treat acute intestinal obstruction caused by Yellowstone, which can significantly control the disease progression and relieve abdominal distention and pain. Kong et al. [22] applied continuous aspiration and infusion of a three-chamber drainage tube combined with somatostatin for acute intestinal obstruction, which can significantly reduce the intestinal lumen pressure. At the same time, it can relieve the blockage of fibrous tissue, improve the gastrointestinal environment, and improve the effective rate of treatment. The results showed that the duration of abdominal distention and abdominal pain was shorter in the former than in the latter. The amounts of gastrointestinal decompression, drainage flow, and abdominal circumference reduction in the former were higher than those in the latter. After treatment, the levels of CRP, IgA, LPS, and FABP in each group were lower than before, and the levels of CRP, IgA, LPS, and FABP in the former group were lower than the latter. The results are basically similar to those of Lin and Kong, suggesting that somatostatin combined with transnasal intestinal obstruction catheterization can effectively relieve gastrointestinal discomfort and reduce the expression of inflammatory factors in patients with acute intestinal obstruction. In the procedure of transnasal intestinal obstruction catheterization, the catheterization has ideal hydrophilicity and bearing capacity, which can suck intestinal contents near the intestinal obstruction and improve the abdominal cavity teeth. At the same time, it can regulate gastrointestinal blood gas circulation and blood transport function and promote obstruction sites unimpeded. Combined use of somatostatin can effectively improve gastrointestinal inflammation, control the expression of CRP, IgA, LPS, FABP, inflammatory response, and gastrointestinal injury, and increase the reduction of gastrointestinal pressure.

Patients with acute intestinal obstruction with advanced gastric cancer often affect treatment compliance due to illness, pain, mental stress, etc. In addition, due to the differences in the degree and constitution of intestinal obstruction, there will be different degrees of discomfort and complications during the treatment, which will affect the therapeutic effect. Nishie et al. [23] treated patients with adhesive small intestinal obstruction with transnasal obstruction catheterization, which can significantly improve clinical efficacy, control postoperative recurrence and adverse reactions, and improve the postoperative survival rate. The results were that after treatment, each group's score on conscious behavior, physiological state, psychological emotion, social role, and special situations was higher than before treatment. The team GIQLI scale score is significantly higher than the control group. After treatment, the effective rate of the study group was significantly higher than the control group. Team postoperative complication rates were significantly lower than the control group. The results were basically similar to those of Nishie, suggesting that the intervention of somatostatin combined with transnasal intestinal obstruction catheter placement for patients with acute intestinal obstruction combined with advanced gastric cancer can effectively improve patients' mental and physical mobility and promote their rapid recovery. The transnasal intestinal obstruction catheter can reach the obstruction site or the accumulation site of intestinal contents along with gastrointestinal peristalsis, which can achieve continuous decompression in the gastrointestinal tract. In addition, through continuous suction of intestinal contents, perfusion of distilled water, etc., can relieve abdominal pressure, adjust the balance of water, electrolyte, acid and base, improve the immune system function, and control the recurrence of the disease. Combined with somatostatin therapy, it can regulate the ability of gastrointestinal gas and fluid accumulation and promote the recovery of gastrointestinal function. At the same time, the gastrointestinal mucosa should be protected as much as possible, and the mucosal permeability should be reduced, so as to achieve a significant therapeutic effect, providing reference and ideas for clinical treatment.

Although the therapeutic effect of this study is significant, there are still some limitations. The limited sample size of this study may affect the accuracy of clinical results to a certain extent. Failure to explore long-term outcomes for patients may affect the credibility of the findings. Therefore, it is necessary to further expand the sample size and extend the follow-up time to explore the general adaptability and long-term safety.

In conclusion, somatostatin combined with transnasal obstruction catheterization for acute intestinal obstruction with advanced gastric cancer can promote early recovery of clinical symptoms, control the expression of CRP, IgA, LPS, and other inflammatory factors, and improve the patient's quality of life. Its safety and feasibility are high, and it has the value of popularization and application.

## Figures and Tables

**Figure 1:** Comparison of serum related indicators ((a): CRP; (b): IgA; (c): LPS; (d): FABP, compared with before treatment and control group, ^*∗*#^*P* < 0.05).

**Figure 2:** 2GIQLI score comparison: (a) conscious behavior; (b) physiological state; (c) psychological mood; (d) social role; (e) special situation, compared with before treatment and control group, ^*∗*#^*P* < 0.05.

**Table 1:** Comparison of gastrointestinal function improvement ($\bar{x}$ ± *s*).

Group	Control group (*n* = 47)	Study group (*n* = 47)
Duration of abdominal distention (h)	43.59 ± 10.25	27.13 ± 8.32^#^
Normal exhaust time (D)	7.03 ± 1.64	4.54 ± 1.24^#^
Gastrointestinal decompression volume (mL)	594.32 ± 105.42	1139.47 ± 153.37^#^
Discharge flow (mL)	337.25 ± 86.89	664.25 ± 112.09^#^
Abdominal circumference reduction (cm)	9.67 ± 2.81	15.38 ± 3.05^#^

Compared with control group, ^#^*P* < 0.05.

**Table 2:** Comparison of serum-related indicators ($\bar{x}$ ± S).

Group	Time	Control group (*n* = 47)	Study group (*n* = 47)
*CRP (mg/L)*	Before the treatment	35.61 ± 7.38	35.62 ± 7.40
	After the treatment	24.69 ± 5.64^*∗*^	14.35 ± 4.32^∗#^

*IgA (g/L)*	Before the treatment	2.19 ± 0.51	2.16 ± 0.52
	After the treatment	1.82 ± 0.45^*∗*^	1.54 ± 0.36^∗#^

*LPS (μmol/L)*	Before the treatment	193.62 ± 24.69	192.84 ± 24.70
	After the treatment	84.59 ± 17.72^*∗*^	41.38 ± 12.34^∗#^

*FABP (ng/L)*	Before the treatment	275.64 ± 22.56	274.95 ± 23.14
	After the treatment	225.86 ± 19.67^*∗*^	175.68 ± 16.35^∗#^

Note, compared with control group, ^#^*P* < 0.05.

**Table 3:** Comparison of GIQLI scores ($\bar{x}$ ± *S*, points).

Group	Time	Control group (*n* = 47)	Study group (*n* = 47)
*Conscious activity*	Before the treatment	16.48 ± 4.23	16.47 ± 4.25
	After the treatment	17.91 ± 4.52^*∗*^	21.50 ± 4.83^∗#^

*Physiological state*	Before the treatment	16.10 ± 3.04	16.11 ± 3.05
	After the treatment	17.32 ± 3.24^*∗*^	19.48 ± 3.34^∗#^

*Psychological mood*	Before the treatment	15.58 ± 3.17	15.59 ± 3.15
	After the treatment	17.64 ± 3.30^*∗*^	20.07 ± 3.46^∗#^

*Social role*	Before the treatment	15.97 ± 3.69	15.93 ± 3.68
	After the treatment	17.68 ± 3.82^*∗*^	20.18 ± 4.10^∗#^

*Special conditions*	Before the treatment	18.59 ± 2.57	18.57 ± 2.60
	After the treatment	19.73 ± 2.61^*∗*^	21.65 ± 2.83^∗#^

Compared with the control group, ^#^*P* < 0.05.

**Table 4:** Comparison of therapeutic effects (cases, %).

Group	Control group (*n* = 47)	Study group (*n* = 47)	*χ* ^2^	*P*
Heal	24 (51.06)	30 (63.83)	—	—
Valid	17 (36.17)	15 (31.91)	—	—
Invalid	6 (12.77)	2 (4.26)	—	—
Therapeutic response rate	87.23%	95.74%	0.924	0.001

**Table 5:** Comparison of incidence of adverse reactions (cases, %).

Group	Control group (*n* = 47)	Study group (*n* = 47)	*χ* ^2^	*P*
Infection	2 (4.26)	0 (0.00)	—	—
Allergic reaction	1 (2.13)	1 (2.13)	—	—
Nausea and vomiting	1 (2.13)	2 (4.26)	—	—
Vertigo	1 (2.13)	0 (0.00)	—	—
Abdominal cavity effusion	2 (4.26)	1 (2.13)	—	—
Incidence of postoperative complications	14.89%	8.51%	2.307	0.019

## Data Availability

The data used to support the findings of this study are available from the corresponding author upon request.
